RETRACTED

# Continual Digital Twin Technology Application on the Construction of English-Chinese Bilingual Teaching Mode

**DOI:** 10.1155/2022/6423550

**Published:** 2022-06-15

**Authors:** Wang Haijie, Zhang Li

**Affiliations:** Western Languages Department, Hebei Institute of International Business and Economics, Qinhuangdao 066311, Hebei, China

## Abstract

This study enhances the conventional English-Chinese bilingual teaching mode by incorporating the continuous digital twin technology into its design. In addition to the typical video and audio transmission teaching functions, the English-Chinese bilingual distant education system also includes a number of interactive capabilities. The approach described in this study is mostly utilized for bilingual instruction in colleges and universities, and the instruction is enhanced by digital twin technology. In this work, the system performance test focuses primarily on the evaluation of teaching quality and teaching satisfaction. Among these are the evaluation of teaching quality by questionnaires, the evaluation of this paper's system by a number of senior teachers, and the calculation of student satisfaction through teaching experiments. The results of the study indicate that the strategy described in this work has a particular effect.

## 1. Introduction

### 1.1. Background

Language, culture, knowledge, careers, and other factors are advancing toward globalization, internationalization, and informationization against the backdrop of economic globalization. The proficient use of English, particularly subject-specific professional English, has evolved into a necessity. However, there are still many unsatisfactory aspects in my country's college English teaching [1]: English teaching still stays on the basis of “grammar translation method,” the classroom teaching method is single, the rhythm is slow, the amount of information is insufficient, and the practice is lacking. In addition, teachers follow the book to “full house,” and students passively accept and lack interest. In the limited classroom teaching time, foreign languages are invaded by their mother tongue and students cannot use English to understand and think communicative skills, which has caused the reality that it is difficult for Chinese students to pass the test in English. As a result, the school must conform to the needs of the times and increase the intensity of education reform in the cultivation of talents in the new century.

### 1.2. Problem Proposal

The proposal and implementation of bilingual teaching are an important measure to truly change the traditional education system and establish new scientific education goals. Bilingual teaching is conducive to absorbing the world's advanced and scientific cultural knowledge to serve my country's economic construction [2], and it is conducive to promoting China's advanced culture and science to the world. The internationalization of higher education is an inevitable requirement of economic globalization. China's accession to the World Trade Organization means that China participates in economic globalization at a deeper level. Humanity's future is bilingual. In the context of economic globalization, a big number of high-level individuals who are skilled in English and master and apply professional knowledge are needed to adapt to and succeed in the international market competition. This puts forward higher requirements for the development of education. At the same time, education also needs to make adjustments in order to meet the needs of the development of the times. Moreover, English is the world language. In order to achieve the internationalization of higher education and enhance the international competitiveness of universities, in addition to curriculum settings that must meet the requirements of the times, the implementation of bilingual teaching is also an effective method [3].

RETRACTED

Science and technological progress depend on education. Educational concepts and instructional content should closely track current knowledge and topic research frontiers to fulfill the country's talent training requirements, so college students can quickly grasp basic professional knowledge and the latest breakthroughs in connected disciplines. Bilingual teaching on campus is a teaching trend. Education internationalization is increasing to connect with the world. China's higher education is more competitive since joining the WTO. Through overseas teaching experience, my country's institutions can be internationally competitive, increase its education position, and train international talents. In order to react to the difficulties of economic globalization and technological change, international sports organizations must grasp professional knowledge, skills, and tactics in English. This is a policy and societal imperative.

At present, the focus of higher education reforms is mainly on two aspects: one is to promote bilingual teaching in education, and the other is to promote the use of information technology in teaching, especially teaching using network technology. Network-assisted teaching is a teaching method based on the integration of information technology (network technology) and subject courses. It is a new type of course teaching task that is combined with the network organically without departing from traditional classroom teaching methods. In bilingual teaching, traditional classroom teaching has been shown to be unable to meet the needs of teaching in terms of modes and methods. The development of a bilingual teaching support system based on WEB is an extension and expansion of conventional bilingual teaching, as well as teaching reform, and it is an inevitable requirement to improve the quality of bilingual teaching. This system takes the syllabus as the goal, uses modern information technology as the means, and takes the convenience of teacher use as the key technology to meet the needs of bilingual education. The development of this system will greatly promote both the learning of students and the teaching of teachers and will help improve the quality of bilingual teaching in an all-round way.

RETRACTED

This article combines the digital twin technology and an intelligent teaching system to improve the English-Chinese bilingual teaching mode and the quality of English-Chinese bilingual teaching.

## 2. Related Work

The basic working principle of the fast Fourier transform algorithm based on frequency domain analysis [4] is to use the fast Fourier transform FFT algorithm to decompose and transform the signal sampled in a whole cycle. Thus, parameters such as the amplitude, frequency, and phase of the fundamental wave and each harmonic may be determined, and the functional equations of the fundamental wave and each harmonic can be solved for their mathematical expressions. The downside of this approach is that the sampled signal must be assured to be within a full cycle, resulting in a considerable delay in the calculated output. With the rapid advancement of chip technology, the processing capability of digital signals is increasing and the calculation speed is accelerating, which drastically reduces the algorithm's latency and accelerates its real-time performance. Nevertheless, when the signal is sampled asynchronously, signal leakage and fence effects must occur. Moreover, the parameters such as amplitude, phase, and frequency calculated by this algorithm have large errors, which cannot guarantee the requirements of signal measurement accuracy [5]. Some scholars at home and abroad have conducted related research on this algorithm. In order to better improve the measurement accuracy of the algorithm, the literature [6] adopted an interpolation algorithm to interpolate and correct the data processed by fast Fourier transform FFT. It is found that the error can be effectively reduced. The literature [7] proposed a Hanning window to truncate the signal to reduce the leakage effect when the signal is truncated, which significantly reduces the calculation error. The literature [8] adopted a windowed single-peak spectral line interpolation correction algorithm, using the highest spectral line near the frequency point to interpolate and correct the phase. It is found that in a small range, the phenomenon of signal spectrum leakage can be effectively suppressed. There are also many scholars in China who conduct a lot of research and analysis. The literature [9] used a Blackman–Nuttall convolution window function. In terms of the sidelobe attenuation of the window function, it is obviously better than the Hanning window, and the error of the corrected data is significantly reduced. The literature [10] used a bimodal spectral line interpolation correction on the FFT processed data. The algorithm uses two spectral lines near the measured frequency point to interpolate and correct them after the weighted average and approximate the corrected data with a function polynomial. The literature [11] overcomes the difficulties of numerical calculations in mathematical calculations, at the same time improved the accuracy of the calculation results and reduced the complexity of the algorithm in time and space.

RETRACTED

With the continuous improvement of the industrial automation level, the requirements for sensor signal acquisition technology are getting higher and higher, no matter in terms of accuracy or speed. With the widespread application of 32-bit single-chip microcomputers, a sensor acquisition system based on a combination of single-chip microcomputers and computers has appeared [12]. This structure is developed from the application field of the compute and is connected to the computer by a 32-bit single-chip microcomputer through a bus. Among them, the function of sensor signal acquisition is the responsibility of the single-chip microcomputer and its interface circuit. The collected data are transmitted to the upper computer through the bus for storage and processing, and the processed results are fed back to the lower computer for related operations so that the upper computer and the lower computer are synchronized [13–15]. The characteristics of the system are the following: ① The system is open source, anyone can develop independently on it to improve the functions of the system. ② When configuring the software and hardware of the computer and the single-chip computer, it is flexible and able to construct a large-scale network monitoring system. ③ The system has high efficiency, makes full use of the resources of the microcontroller and computer, and does not occupy the memory of the CPU, but the cost is high [14–16].

## 3. Signal Processing Algorithm Based on Digital Twin Technology

The process of restoring student image information is to diffuse and fill the damaged area with information from the undamaged area in the image, as shown in Figure 1. Among them, *I* is the entire image, and Ω is the damaged area.

RETRACTED

The essence of visual information restoration for students is to diffuse and fill the damaged area with information from the undamaged area. However, because there is insufficient information to guarantee the validity and uniqueness of the restored information, the restoration of student image information is, from a mathematical perspective, a grave issue [17]. The process of populating the image with information is completed recursively. The specific formula of the algorithm is as follows:

(1) $$\begin{array}{c} I^{n+1}\left(i,j\right)=I^{n}\left(i,j\right)+\Delta tI_{t}^{n}\left(i,j\right),\;\forall \left(i,j\right)\in \Omega . \end{array}$$

Among them, *n* represents the number of recursions in the repair process, (*i*, *j*) represents the horizontal and vertical coordinates of the pixel *I*_*t*_^*n*^(*i*, *j*), Δ*t* represents the rate of image improvement after each recursion, and *I*_*t*_^*n*^(*i*, *j*) represents the amount of further improvement on *I*^*n*^(*i*, *j*). The expression is

(2) $$\begin{array}{c} I_{t}^{n}\left(i,j\right)=\left[\delta {\overset{⟶}{L}}^{n}\left(i,j\right)\cdot \frac{\overset{⟶}{\overset{⟶}{N}}\left(i,j,n\right)}{\left|\overset{⟶}{N}\left(i,j,n\right)\right|}\right]\left|\nabla I^{n}\left(i,j\right)\right|. \end{array}$$

Among them, $\overset{⟶}{N}/\left|\overset{⟶}{N}\right|$ is the isoilluminance line direction and generally takes the orthogonal direction of the image gradient vector ∇*I*^*n*^, which means that the information propagates into the damaged area, *L*^*n*^ is the image smoothness measurement, which is usually calculated by the Laplacian operator; $\delta {\overset{⟶}{L}}^{n}$ represents the amount of change of the inward propagation information *L*^*n*^, and when the algorithm reaches a steady state, *I*^*n*+1^(*i*, *j*) ≈ *I*^*n*^(*i*, *j*).

The mathematical model of total variation (TV) is applied to the restoration of student image information. The algorithm uses the variational method to solve the energy minimization equation to achieve the restoration of the damaged area of the image. The specific formula is as follows:

(3) $$\begin{array}{c} J\left(I\right)=\int_{E\cup \Omega }\left|\nabla I\right|\text{dx dy}+\frac{\lambda }{2}\int_{E}\left|I-I^{0}\right|\text{dx dy}. \end{array}$$

Among them, Ω is the area to be repaired, *E* is the intact area surrounding Ω, *λ* is the Lagrangian operator, *I* is the pixel information of the repaired image, and *I*^0^ is the pixel information of the known part of the unrepaired image. At the same time, the time variable *t* is introduced, and the energy descent equation is solved by the steepest descent method, which is expressed as follows:

(4) $$\begin{array}{c} \frac{\partial I}{\partial t}=\nabla \left[\frac{\nabla u}{\left|\nabla u\right|}\right]+\lambda_{D}\left(I^{0}-I\right). \end{array}$$

Among them, when (*x*, *y*) ∈ *E*, *λ*_*D*_=*λ*, and when (*x*, *y*) ∈ Ω, with the change of time *t*, when ∂*I*/∂*t*⟶0, the minimum value of I is obtained.

RETRACTED

The main advantage of the TV model compared with the BSCD model is that the model can maintain the edge and has good stability [18, 19]. The main disadvantage is that this model destroys the connection principle in visual theory. As shown in Figure 2, it represents the structural width of the target and the width of the area to be repaired. Regardless of the ratio of the sum, Figure 2(b) is considered to be the best repair effect according to human visual psychology. However, for the TV model, when *w*_1_ < *w*, the repair effect is 2(b), and when *w*_1_ > *w*, the repair effect is shown in Figure 2(c). This destroys the principle of connectivity.

In order to improve the above shortcomings of the TV model, Chan and Shen [20] proposed a Curvature Driven Diffusions (CDD) model [20]. In this model, Chan and Shen [20] introduced the curvature *k* into the model and defined the conduction function as follows:

(5) $$\begin{array}{c} u=\frac{g\left(\left|k\right|\right)}{\left|\nabla I\right|},\\ g\left(k\right)=\left\{\begin{array}{cc} 0, & k=0,\\ \infty , & k=\infty ,\\ N, & 0<k<\infty . \end{array}\right. \end{array}$$

Among them, *k*=div[∇*I*/|∇*I*|] is the curvature, and *N* is a finite number greater than zero. Because of this choice, the diffusion at the large curvature becomes stronger, and the diffusion at the small curvature gradually disappears. Therefore, the CDD model can be defined as follows:

(6) $$\begin{array}{c} \frac{\partial I}{\partial I}=\text{div}\left[\frac{g\left(\left|k\right|\right)}{\left|\nabla I\right|}\nabla I\right]. \end{array}$$

The Mumford–Shah model was first used for image segmentation and image denoising. Later, Tsai and Chan et al [21]. introduced the model to the field of student image information restoration. The basic idea of the algorithm is to minimize the following energy function:

(7) $$\begin{array}{c} J\left(u,\Gamma ,\Omega \right)=\frac{r}{2}\int_{I/\Gamma }{\left|\nabla u\right|}^{2}\text{dx}+\alpha j\left(\Gamma \right)+\frac{\lambda }{2}\int_{I/\Omega }{\left(u-u^{0}\right)}^{2}\text{dx}. \end{array}$$

Among them, *I* represents the entire image, Γ represents the edge set of the image, *l*(Γ) represents the length of Γ, Ω represents the area to be repaired, *u* represents the pixel value of the repaired image, *u*^0^ represents the pixel value of the intact area of the image, and *α*, *λ*, and *γ* represent weights. When the solution of the above equation is denoted as *μ*_Γ_, the variation of the energy functional *J*(*u*, Γ, Ω) is the following:

(8) $$\begin{array}{c} \gamma \Delta u+\lambda_{\Omega }\left(\chi \right)\left(u^{0}-u\right)=0,\frac{\chi \in I}{T}. \end{array}$$

Corresponding to *J*(*u*, Γ, Ω), the gradient of Γ is reduced to infinitesimal:

(9) $$\begin{array}{c} \frac{\text{dx}}{\text{dt}}=\left[ak+{\left[\frac{\lambda }{2}{\left|\nabla \mu_{\Gamma }\right|}^{2}+\frac{\lambda_{\Omega }}{2}{\left(\mu_{\Gamma }-u\right)}^{2}\right]}_{\Gamma }\right]\overset{⟶}{n}. \end{array}$$

Among them, *x* represents the edge pixel, $\overset{⟶}{n}$ represents the normal vector at *x*, and the symbol [*f*]_Γ_ is the following:

(10) $$\begin{array}{c} {\left[f\right]}_{\Gamma }\left(x\right)=\underset{x⟶0^{+}}{\lim}\left(f\left(x+\Gamma \overset{⟶}{n}\right)-f\left(x-\Gamma \overset{⟶}{n}\right)\right). \end{array}$$

The advantage of the Mumford–Shah model is low-computational complexity, but because the Mumford–Shah model minimizes the edge length. Therefore, the repaired edge is directly connected to the existing edge, which will result in a more obvious angle at the edge connection instead of a smooth curve.

RETRACTED

The Criminisi algorithm can be summarized as the following steps:

(1) Determine the priority coefficient of the sample block at the edge of the damaged area. The repair sequence of the pixels to be repaired at the edge of the damaged area directly affects the quality of the final repair effect, so it is very important to choose an appropriate priority coefficient during the repair process. As shown in Figure 3, point *p* is any point on the edge *α*Φ of the area to be repaired, and Ψ_*p*_ is the block to be repaired with *p* as the center. *C*_*p*_′ represents the confidence factor of the block Ψ_*p*_ to be repaired, and Ψ_*p*_ is the ratio of intact pixels to the total number of pixels in the block. It can be seen from the definition of *C*_*p*_′ that the larger the *C*_*p*_′, the more known information contained in the block to be repaired, and it should be repaired first. *D*_*p*_ represents the structure factor of the block to be repaired, that is, the structure information of the block to be repaired Ψ_*p*_, and its definition is shown in formula (12). It can be seen from the definition of *D*_*p*_ that the larger the structure factor, the stronger the structure of the block to be repaired, and it should be repaired first. According to the above analysis, the priority coefficient of the block to be repaired is defined as follows:
  (11) $$\begin{array}{c} P_{p}=C_{p}^{\prime }\cdot D_{p}, \end{array}$$
  (12) $$\begin{array}{c} C_{p}^{\prime }=\frac{\sum_{q\in \Psi \cap \bar{\Omega }}C_{q}}{\left|\Psi_{p}\right|},D_{p}=\frac{\left|\nabla {Ι}_{p}^{⊥}\cdot n_{p}\right|}{\alpha }. \end{array}$$
Among them, |Ψ_*p*_| represents the total number of pixels contained in Ψ_*p*_, $\bar{\Omega }$ represents the intact area of the image, $\Psi_{p}\cap \bar{\Omega }$ represents the intact pixels in the block Ψ_*p*_ to be repaired, and *C*_*q*_ represents the confidence of any point *Ψq* on the image. In addition, *α* is a normalization factor. If the value of each component of the image is 255, then *α* = 255. The purpose is to make 0 ≤ *D*_*p*_ ≤ 1, that is, to ensure that *C*_*p*_′ and *D*_*p*_ have the same degree of influence on the priority coefficient. *n*_*p*_ is the normal vector of the tangent line at point *p*, and ∇Ι_*p*_^⊥^ represents the vertical direction of the gradient direction at point *p*, that is, the direction of the isoilluminance line. The specific calculation formula is as follows:
  (13) $$\begin{array}{c} \nabla {Ι}_{p}^{⊥}=\frac{\left(-I_{y}\left(p\right),I_{x}\left(p\right)\right)}{\sqrt{I_{x}{\left(p\right)}^{2}+I_{y}{\left(p\right)}^{2}}}. \end{array}$$
Among them, *I*_*x*_(*p*) and *I*_*y*_(*p*) represent the partial differentials of point *p* in the *x* and *y* directions, respectively.
Generally, *C*_*q*_ is initialized as follows:
  (14) $$\begin{array}{c} C_{q}=\left\{\begin{array}{cc} 0, & \forall q\in \Omega ,\\ 1, & \forall q\in \bar{\Omega }. \end{array}\right. \end{array}$$
The confidence level *C*_*p*_′ represents the proportion of known pixels in the block Ψ_*p*_ to be repaired. The more intact pixels in Ψ_*p*_, the greater *C*_*p*_′. Therefore, for each point in the area to be repaired, the closer to the center area, the smaller the value of the confidence *C*_*p*_′, so to a certain extent, it is ensured that the repair sequence gradually deepens from the outside to the center of the damaged area.
*D*_*p*_ represents the intensity of the isoilluminance line at point *p*. It can be seen from formula (13) that the size of *D*_*p*_ is determined by the angle |∇Ι_*p*_^⊥^ · *n*_*p*_| between the intensity of the isoilluminance at point *p* and the normal vector at point *p*. |∇Ι_*p*_^⊥^ · *n*_*p*_| reflects the consistency of the two vector directions. The smaller the angle between the two vectors, the larger the value, the larger the value of *D*_*p*_, the richer the structural information in Ψ_*p*_, and the higher the calculated priority, then Ψ_*p*_ should be repaired first. Conversely, the smaller the value of *D*_*p*_, the less structure information in Ψ_*p*_, and the lower the calculated priority.
It can be seen from the above analysis that the priority coefficient *D*_*p*_ reflects both the confidence of the block to be repaired and the structural strength of the image. The order of restoration of student image information determined by this coefficient not only achieves priority restoration of areas with a lot of known information to ensure the correct diffusion of information, but also achieves priority restoration of structural parts, which makes the restored image remain visually connected, and effectively avoids mismatches and faults that may occur during the restoration process.
(2) Find the best matching block
After finding the block to be repaired with the largest priority coefficient through step 1, we search for the intact sample block that best matches the block in the intact area of the image and fill the damaged points in the block to be repaired with the pixel information of the block. After that, we select the rectangular block Ψ_*p*_ with the largest priority coefficient and centered on *p* to be repaired and find the best matching sample block Ψ_*p*_ in the intact information area, so that it satisfies the relationship:
  (15) $$\begin{array}{c} \Psi_{p}=\arg\min\Psi_{q^{\prime }\subset \Gamma }d\left(\Psi_{p},\Psi_{q^{\prime }}\right),\\ d\left(\Psi_{p},\Psi_{q^{\prime }}\right)=\sum_{\alpha \in \Psi_{p},b\in \Psi_{p}}\sqrt{{\left(R\left(\alpha \right)-R\left(b\right)\right)}^{2}+{\left(G\left(\alpha \right)-G\left(b\right)\right)}^{2}+{\left(B\left(\alpha \right)-B\left(b\right)\right)}^{2}}. \end{array}$$
Among the blocks to be matched, the block to be matched with the smallest value of *d* is found, and this block is the optimal matching block of the block Ψ_*p*_ to be repaired.
(3) Information filling
Through the above method, the propagation of the pixel information of the intact area of the image to the pixel information of the area to be repaired can be completed, and the structure and texture information of the intact area can be diffused to the damaged area.
(4) Update confidence
It can be seen from the definition of confidence that the confidence of each point in the area to be repaired is all initialized to 0, and when the missing information in Ψ_*p*_ is filled with new information, the confidence of the filled pixel needs to be updated at the same time. The confidence level *C*_*q*_ is updated according to the following formula:
  (16) $$\begin{array}{c} C_{q}=C_{p}^{\prime }\;\forall q\in \Psi_{p}\cap \Omega . \end{array}$$

That is, the confidence of the damaged pixel that is filled is replaced by the confidence of the block where the point is located.

RETRACTED

## 4. Construction of English-Chinese Bilingual Teaching Model Based on Digital Twin Technology

Technical difficulty and research focus on the full localization or un-lcode internationalization of the original ANSI standard system. On this foundation, English-Chinese bilingualization and dynamic interface switching are achieved.

According to the requirements of the C/S development model, in the VC and Delphi development environment required by the system, a thorough in-depth analysis of the ANSI standard SkyClass modern distance learning system structure and source code must be made, and the following aspects of development work should be done [21–23]: ① Pass the secondary development and transformation of the original system and the improvement of the classroom service center module (Server) with management and control of classroom and user processes and the intermediate station service module MultiControlUnit (MCU) with the function of one-to-many forwarding of classroom information, make these modules support The normal display of English-containing complex characters using the Unicode standard and the normal communication between such language information and the client. ② Through the secondary development and improvement of the two client modules of the original system, teacher's teaching terminal and student listening terminal, make these modules support the use of Unicode standard English-containing complex text and realize bilingual electronic pointers and teacher–student interactive dialogue. ③ Through the secondary development of all modules of the original system, from the entire system user interface and kernel related code Angle, redesign and implement, and launch a new version of each module with English-Chinese bilingual user interface. ④ Take the most reliable and fastest solution to realize the bilingualization of the entire system and the dynamic switching function of the English-Chinese bilingual interface during runtime. ⑤ Through the use of software engineering-related testing methods to debug and improve the entire English-Chinese bilingual distance education system, the products are put on the market.

The system should consist of four principal modules: the classroom service center (Server), the one-to-many multicast multipoint control unit (MCU), the multimedia teaching terminal (Teacher), and the multimedia listening terminal (Listener) (Student). The Server and MCU programs are installed independently on fixed network machines, the Teacher program is installed on the computer of the networked teacher, and the student application is installed on the computer of the networked student. The final three modules must be logged into the server application prior to instruction. Then during the lecture period, the MCU uses a one-to-many rebroadcast method to stream the computer screen, video, and audio information of the lecture section to each student's listening terminal to realize the synchronized network multimedia teaching by the famous teacher. The overall simple framework of the system is shown in Figure 3:

In addition to the traditional video and audio transmission teaching functions, the English-Chinese bilingual distance teaching system also has certain interactive functions. The system structure is divided into four subsystems, as shown in Figure 4.

RETRACTED

The network topology design of the English-Chinese bilingual distance teaching system is as follows Figure 5:

According to the system architectural diagram's functions and communication relationships, the system can be separated into four subsystem modules: the classroom service center, the multipoint forwarding module, the teacher teaching terminal, and the student listening terminal. The functions of these subsystem modules are allocated as follows Figure 6:

The topology of the network is the first step in the design plan, and it is also a very important step. The core layer is composed of two Layer 3 switching routers Huawei 6503. The switches are connected to each other through a 1000 M link, and each is connected to the campus network backbone through a 1000 M link (Figure 7). It can share the load equally and back up each other. Outside the switch core, the stacks of multimedia classrooms (BS450/BS350/BS303) are connected radially. It can be 2–4 sets to provide about sixty 10/100 M Ethernet ports to connect sixty multimedia PCs.

Logical design is to convert the data pattern generated by conceptual design into a data pattern represented by logical data. The logical structure of a relational model is a collection of relational patterns. Converting the E-R diagram into a relational model is actually to transform the entity, the attributes of the entity, and the connection between the entities into a relational model.

The logical design structure of the MySQL database is shown in Figure 8.

JSP is by extension. JSP file to achieve, a JSP is equivalent to an executable file, so it must be placed in a directory with executable permissions on the Web server. When the browser requests the JSP file from the WebServer for the first time, the WebServer starts to call the JSP. The JavaServlet engine compiles the requested. JSP file into a Servlet and then dynamically generates an HTML page and sends it to the browser. In the future, when the browser requests to call for the JSP file from the WebServer, there is no need to recompile, as long as the existing Servlet is executed.

RETRACTED

## 5. System Test

This study combines a digital twin technology with an English-Chinese bilingual teaching mode to create a system, and then analyzes the system's performance using a performance test. The approach described in this study is mostly utilized for bilingual instruction in colleges and universities, and the instruction is enhanced by digital twin technology. In this work, the system performance test focuses primarily on the evaluation of teaching quality and teaching satisfaction. Among them, the evaluation of teaching quality is carried out by means of questionnaires, the system of this paper is evaluated by a number of senior teachers, and the satisfaction is calculated by means of teaching experiments. The final results are shown in Tables 1 and 2 and Figures 9 and 10.

From the above analysis, it can be seen that the English-Chinese bilingual teaching system based on the digital twin technology constructed in this paper has a good teaching effect and has a certain degree of humanity, which can meet the various needs of users.

## 6. Conclusion

The creation of a bilingual teaching quality assurance system in colleges and universities must follow the relevant characteristics and rules, reflect the distinctiveness of bilingual teaching, and be very relevant. Bilingual teaching should reflect bilingual teaching's guiding ideology, talent training objectives, majors, courses, teachers, teaching quality management, and monitoring.

A bilingual teaching quality assurance system must be built based on these characteristics. Only a quality assurance system based on bilingual teaching characteristics and the status quo can adapt to the actual situation of bilingual teaching in colleges and universities and guarantee and improve its quality. This paper creates a digital-twin-based English-Chinese teaching system. This approach improves English-Chinese bilingual instruction.

## Figures and Tables

**Figure 1:** Schematic diagram of student image information restoration.

**Figure 2:** Schematic diagram of the principle of visual connection.

**Figure 3:** The overall framework of the English-Chinese bilingual teaching system.

**Figure 4:** Use case diagram of bilingual distance teaching system. (a) Client. (b) Server.

**Figure 5:** Network topology structure of English-Chinese bilingual distance teaching system.

**Figure 6:** Schematic diagram of module functions of English-Chinese bilingual distance education system.

**Figure 7:** Network structure diagram of teaching system.

**Figure 8:** The logical design structure of the database.

RETRACTED

**Figure 9:** Statistical diagram of teaching evaluation effect.

**Figure 10:** Statistical diagram of system user satisfaction survey.

**Table 1:** Statistical table of teaching evaluation effect.

Num	Teaching evaluation
1	89.20
2	86.47
3	81.12
4	92.03
5	89.76
6	89.81
7	84.23
8	90.06
9	89.54
10	91.53
11	90.76
12	82.99
13	86.31
14	92.90
15	86.34
16	88.03
17	86.76
18	81.64
19	82.00
20	90.84
21	87.98
22	85.92
23	88.93
24	83.68
25	90.72
26	81.56
27	91.06
28	87.38
29	84.96
30	87.79
31	90.08
32	83.13
33	88.62
34	84.31
35	82.70
36	91.89
37	82.97
38	81.38
39	83.27
40	86.73
41	92.15
42	81.49
43	92.68
44	85.15
45	92.27
46	87.55
47	82.13
48	89.90
49	86.20
50	81.28
51	86.60
52	85.89
53	81.42
54	88.81
55	85.92
56	86.03
57	83.69
58	90.93
59	84.41
60	87.84
61	82.06
62	90.30
63	86.09
64	87.54
65	89.77
66	90.53
67	81.43
68	91.35
69	82.80
70	81.39
71	91.81
72	92.38
73	83.27
74	86.78
75	86.19

**Table 2:** Statistical table of system user satisfaction survey.

Num	Teaching evaluation
1	89.20
2	86.47
3	81.12
4	92.03
5	89.76
6	89.81
7	84.23
8	90.06
9	89.54
10	91.53
11	90.76
12	82.99
13	86.31
14	92.90
15	86.34
16	88.03
17	86.76
18	81.64
19	82.00
20	90.84
21	87.98
22	85.92
23	88.93
24	83.68
25	90.72
26	81.56
27	91.06
28	87.38
29	84.96
30	87.79
31	90.08
32	83.13
33	88.62
34	84.31
35	82.70
36	91.89
37	82.97
38	81.38
39	83.27
40	86.73
41	92.15
42	81.49
43	92.68
44	85.15
45	92.27
46	87.55
47	82.13
48	89.90
49	86.20
50	81.28
51	86.60
52	85.89
53	81.42
54	88.81
55	85.92
56	86.03
57	83.69
58	90.93
59	84.41
60	87.84
61	82.06
62	90.30
63	86.09
64	87.54
65	89.77
66	90.53
67	81.43
68	91.35
69	82.80
70	81.39
71	91.81
72	92.38
73	83.27
74	86.78
75	86.19

## Data Availability

The data used to support the findings of this study are included within the article.
